# Research on Face Recognition Algorithm Based on Image Processing

**DOI:** 10.1155/2022/9224203

**Published:** 2022-03-18

**Authors:** Yan Sun, Zhenyun Ren, Wenxi Zheng

**Affiliations:** College of Information and Communication Engineering University, Harbin 150001, Heilongjiang, China

## Abstract

While network technology is convenient for our daily life, the problems that are exposed are also endless. The most important thing for everyone is information security. In order to improve the security level of network information and identify and detect faces, the method used in this paper has improved compared with the traditional AdaBoost method and skin color method. AdaBoost detection is performed on the image, which reduces the probability of false detection. The experiment compares the experimental results of the AdaBoost method, the skin color method and the skin color + AdaBoost method. All operations in the KPCA and KFDA algorithms are performed by the inner product kernel function defined in the original space, and no specific non-linear mapping function is involved.The full name of KPCA is kernel principal component analysis. The full name of KFDA is kernel Fisher discriminant analysis. Combining the zero-space method kernel discriminant analysis method improves the ability of discriminant analysis to extract non-linear features. Through the secondary extraction of PCA features, a better recognition result than the PCA method is obtained. This paper also proposes a zero-space based Fisher discriminant analysis method. Experiments show that the zero-space-based method makes full use of the useful discriminant information in the zero space of the intraclass dispersion matrix, which improves the accuracy of face recognition to some extent.If you choose the polynomial kernel function, when *d* = 0.8, KPCA has a higher recognition ability. When *d* = 2, the recognition rate of KFDA and zero space-based KFDA is the largest. For polynomial functions, in general, *d* = 2.

## 1. Introduction

In recent years, especially in areas where some terrorist attacks have been raging, various types of information identification and detection have become of great importance. Due to their own broad application areas, as well as false detections and missed inspections, it will cause our public safety. Great threats, these characteristics make information detection and recognition become more important. After the continuous exploration and practice of human beings, the emergence of biometric-based face detection and recognition technology has attracted the attention of most people. Because the biological signs are not interfered by external conditions, the formation itself is also determined by the individual's genes. The individual's genes themselves are unique and cannot be forged, and are well received by everyone. No matter which type of biological certificate, it has its own uniqueness. These uniquenesses are inherently formed by individuals and cannot be trained and forged. Later, the more mature computer image processing technology can basically detect and identify these biological signs.

Although humans can detect and identify a person from the face without difficulty in the case of great changes in expression, age, or hairstyle, it is very difficult to establish a system that can fully automate face recognition. It involves a lot of knowledge in pattern recognition, image processing, computer vision, psychology, etc., and is closely related to the identification methods based on other biometrics and computer human-computer perception interaction. At this time, computer vision technology began to enter people's field of vision as the world developed.

In order to improve the security level of network information, the face is identified and detected. In this paper, the combination of skin color and AdaBoost is used. The previous experiments and the analysis of skin color features can eliminate the complex background of nonface and perform AdaBoost detection on images. All operations in the KPCA and KFDA algorithms are performed by the inner product kernel function defined in the original space, and no specific non-linear mapping function is involved. This is the core technique of the kernel learning method. The KPCA and KFDA algorithms can be described in the same framework by constructing a corresponding linear feature space, then projecting the image into this linear space and using the resulting projection coefficients as the identified feature vector.

The introduction part of the article explains the research background and significance of the article and the research status at home and abroad. The method part describes the concept and algorithm of face detection and recognition model. The experimental part describes the data source and parameters. Conclusion The experimental data are analyzed in the Discussion section.

## 2. Literature Review

Based on the uniqueness and advancement of face detection and recognition technology, many research teams at home and abroad have begun in-depth research. In [1], the author proposes a new face SR method based on Tikhonov regularized neighborhood representation (TRNR). It can overcome the technical bottleneck of the patch representation scheme in the traditional neighbor-embedded image SR method. In [2], the authors evaluated methods using automated face detection techniques to help estimate site use for two chimpanzee communities trapped by cameras. The authors used a traditional manual inspection lens as a baseline to analyze the basic parameters specific to the change to evaluate the performance and practical value of chimpanzee face detection software. In [3], the author describes an automatic parking system that includes a camera mounted at the entrance/exit of the parking lot. If the camera keeps getting frames and detects faces, register them in the database. When the driver leaves, the facial image is captured again at the exit of the parking lot and compared in the database to arrive at the identity. In [4], the author first used the recently introduced 300 VW benchmark to fully evaluate the most advanced deformable face tracking pipeline. Afterwards, many different architectures were evaluated, focusing on the task of online deformable face tracking. In particular, the authors compared the following general strategies: (a) universal face detection plus general facial landmark positioning, (b) universal model free tracking plus generic facial landmark positioning, and (c) mixed state of use state art face detection, model free tracking and facial landmark positioning technology. In [5], the authors propose a method of learning salient features that responds only in the face area. Based on the salient features, the authors have also designed a joint pipeline for detecting and recognizing faces as part of the human-computer interaction (HRI) system of SRU robots. In the experiment, the article analyzes the influence of the saliency term on facial verification and the ability to discriminate against the significant features of LFW. And the experimental results of FDDB verify the effectiveness of the proposed method in face detection. In [6], the author solves these problems by proposing a new video steganography method based on Kanade-Lucas-Tomasi (KLT) tracking using Hamming codes (15, 11). Experimental results show that the method achieves higher embedding capacity and better video quality. In addition, compared with the prior art methods, the proposed algorithm improves the security and robustness of the face detection method. In [7], the authors propose a face recognition system based on low-power convolutional neural network (CNN) for user authentication in smart devices. The system consists of two chips: an always-on function CMOS image sensor (CIS) for imaging and face detection and a low-power CNN processor (CNNP) for face verification (FV). The results of the study show that the function CIS integrated with the FD accelerator can realize event-driven chip-to-chip communication of the face image only when there is a face.

In order to deeply study the characteristics and advancement of computer vision technology, many research teams at home and abroad have applied computer vision technology in different fields. In [8], the author applies computer vision technology to deep learning, and the article briefly outlines some of the most important deep learning programs used in computer vision problems. The authors briefly introduce their history, structure, strengths and limitations, then describe their application in various computer vision tasks, and briefly outline the future direction of designing deep learning solutions for computer vision problems and the challenges involved. In [9], the author applies computer vision technology to image classification, describing the steps involved in quantifying microscopic images and the different methods for each step. The authors used modern machine learning algorithms to classify, cluster, and visualize cells in HCS experiments. In addition to classification or clustering tasks, machine learning algorithms that learn feature representation have recently advanced the state of the art in several benchmarking tasks in the computer vision community. In [10], the author applied computer vision technology to the field of object recognition. Research shows that X-ray test research and development is exploring new methods based on computer vision that can be used to help operators. The article attempts to contribute to the field of object recognition in X-ray testing by evaluating different computer vision strategies proposed in the past few years. For each method, the author provides the results of the experiment displayed on the same database. In [11], the author applied computer vision technology to machine learning, especially support vector machine training, using 26 of the most common tree species in Germany as test cases, classifying specimen images, ideally at the species level. In [12], the author applied computer vision technology to cell segmentation and feature extraction. The authors outline common computer vision and machine learning methods for generating and classifying phenotype profiles, and the need for effective computational strategies for analyzing large-scale image-based data is increasing. Computer vision methods have been developed to aid in phenotypic classification and clustering of data acquired from biological images. In [13], the author applied computer vision technology to visual inspection systems, introduced a vision system for automatic measurement and detection of most types of threads, and developed many image processing and computer vision algorithms to analyze captured. In [14], the authors applied computer vision techniques to type annotations, describing the types of annotations that computer vision researchers use to crowdsource collection, and how they ensure that the data is of high quality while minimizing annotation work. Finally, the author summarizes the future of crowdsourcing in computer vision.

In [15], elated researchers have proposed a powerful framework, named Kernel-norm-based adaptive occlusion dictionary learning, for face recognition with illumination changes and occlusions. Experiments on multiple public datasets show that the NNAODL model can achieve better results than classical methods in the presence of occlusion and illumination changes. In [16], elated researchers propose a novel coupled similarity reference encoding model for age-invariant face recognition by combining nonnegatively constrained reference encoding with coupled similarity measure. Experiments using deep features are performed and high recognition rates are achieved, which shows that the model can be combined with deep networks for better results. In [17], the authors perform some implementations and comparisons of classifiers and 2D sub-space projection methods for face recognition problems. Experimental results show that using these feature matrices with CMA, SVM and CNN in classification problems is more beneficial than using raw pixel matrices in terms of processing time and memory requirements. In [18], Most of the content consists of three parts, namely specific face representation, feature extraction and classification. The face representation represents how the face is displayed and determines the progressive algorithm for detection and recognition. Evaluate face recognition, which considers shape and texture data to talk to images based on local binary patterns for personal free face recognition. In [19], the authors aim to construct facial patterns stored in a digital image database. The process of pattern construction and face recognition starts with an object in the form of a face image, side detection, pattern construction until the similarity of face patterns can be determined, and then face recognition. In this study, a program was designed to test some samples of face data stored in a digital image database so that it could provide similarity of observed face patterns and introduced them using PCA.

## 3. Method

### 3.1. Face Detection and Recognition Model Based on DeepID

#### 3.1.1. Network Structure

The network structure of the Deep ID network is similar to the most basic convolutional neural network. In the Deep ID network structure, the main role of the convolutional network is to classify trained faces. The convolutional network here consists of 4 convolutional layers and 3 pooling layers, and the characteristics of the samples are represented by the last layer in the network. Using a picture as the input of the Deep ID network, the low-level features of the picture are extracted by the lower layer network and calculated layer by layer by convolution, so that the number of extracted features is gradually reduced, and the global structure of the network structure is enhanced. Sex, and can form advanced features in the top-level network structure. The Deep ID network will eventually output an advanced vector of dimension 160, which is highly dense and contains a wealth of authentication information that can be used directly for identification.

#### 3.1.2. Calculation Process

As mentioned before, the network structure of Deep ID includes 4 convolutional layers and 3 pooling layers. Among them, after the first three convolution layers, there is a pooling layer. Behind the fourth convolutional layer, the structure implementation is directly connected to the fully connected layer and through this layer forms an output layer and features for classification. The input picture is divided into categories such as scale, channel, range, etc., and the training process of each vector is relatively independent. Finally, all vectors are connected to obtain the final vector.

#### 3.1.3. Joint Bayesian Model

The joint Bayesian model is also widely used in the field of face recognition. The idea of joint Bayesian model comes from Bayesian face recognition, which mainly consists of dividing a face into two parts, one part is human and human. The difference between the parts is the difference of the individual itself, such as the difference caused by external conditions such as expressions and angles. Then, there are

(1) $$\begin{array}{c} x=\mu +\varepsilon . \end{array}$$

In the formula, *μ* ∝ *N*(0, *S*_*μ*_), represents the difference between people, that is, external differences; *ε* ∝ *N*(0, *S*_*ε*_), represents the difference of the individual itself due to other factors, that is, internal differences. Also assume that both parts are subject to a Gaussian distribution. And by calculating the covariance of the two parts, you can get

(2) $$\begin{array}{c} \sum_{I}=\left[\begin{array}{cc} S_{\mu }+S_{\varepsilon } & S_{\mu }\\ S_{\mu } & S_{\mu }+S_{\varepsilon } \end{array}\right],\\ \sum_{E}=\left[\begin{array}{cc} S_{\mu }+S_{\varepsilon } & 0\\ 0 & S_{\mu }+S_{\varepsilon } \end{array}\right]. \end{array}$$

At this point, the EM iteration of the above formula can get the similarity between the two:

(3) $$\begin{array}{c} r\left(x_{1},x_{2}\right)=\log\frac{P\left(x_{1},x_{2}|H_{I}\right)}{P\left(x_{1},x_{2}|H_{E}\right)}. \end{array}$$

### 3.2. AdaBoost Face Recognition Algorithm Based on Skin Color Segmentation

#### 3.2.1. Color Space

The RGB color space is a color space established by using three kinds of monochromatic light of red (700.0 nm), green (546.1 nm), and blue (453.8 nm) as a coordinate system. According to the principle of three primary colors, in the RGB color space, any color light *F* can be expressed as

(4) $$\begin{array}{c} F=R\left(r\right)+G\left(g\right)+B\left(b\right). \end{array}$$

The RGB color space is based on a Cartesian coordinate system. The three axes of the three-dimensional space correspond to the three primary colors respectively. The coordinate origin corresponds to black, and the corresponding three components *R*, *G*, and *B* are zero. The origin diagonal corresponds to white, and the corresponding three components *R*, *G*, and *B*. The maximum, the three components of the two points on the line *R*, *G*, *B* are equal, corresponding to the gray pixel points, that is, the gray line. The remaining three vertices of the cube correspond to cyan at *R* = 0, purple at *G* = 0, and yellow at *B* = 0. In RGB space, if the value of two pixel points [*R*_1_, *G*_1_, *B*_1_], [*R*_2_, *G*_2_, *B*_2_] are proportional, i.e.,

(5) $$\begin{array}{c} \frac{R_{1}}{R_{2}}=\frac{G_{1}}{G_{2}}=\frac{B_{1}}{B_{2}}. \end{array}$$

The above formula shows that such proportional points have the same color and different brightness, and by normalization, the chrominance components can be removed to obtain the [*r*, *g*, *b*] space, namely,

(6) $$\begin{array}{c} \left\{\begin{array}{c} r=\frac{R}{R+G+B},\\ g=\frac{G}{R+G+B},\\ b=\frac{B}{R+G+B}. \end{array}\right.. \end{array}$$

#### 3.2.2. Skin Color Segmentation

According to the skin color samples in the YCrCb space, the mean value *C*_*b*_, the mean *m* of the *C*_*r*_, and the covariance matrix *C* are calculated by the following formula to obtain

(7) $$\begin{array}{c} {\bar{C}}_{b}=\frac{1}{N}\sum_{i=1}^{N}C_{b_{i}},\\ {\bar{C}}_{r}=\frac{1}{N}\sum_{i=1}^{N}C_{r_{i}}. \end{array}$$

The number of skin color pixels counted by *N* in the above two formulas. Finally, the Gaussian skin color model is defined by the elliptic Gauss joint probability density function:

(8) $$\begin{array}{c} P\left(x|\text{skin}\right)=\frac{1}{2\pi C^{1/2}}\exp\left[-\frac{1}{2}{\left(x-m\right)}^{T}C^{-1}\left(x-m\right)\right], \end{array}$$

where *x* is the color vector, *m* and *C* are the average vector and the covariance matrix, respectively. The probability of the function *P*(*x*|skin) is the skin color similarity of each pixel, which can be used to determine whether it is skin color. Finally, through the threshold setting, an image of the skin color segmentation is obtained. The mean and variance are

(9) $$\begin{array}{c} m={\left(117.43,156.60\right)}^{T},\\ C=\left[\begin{array}{cc} 160.13 & 12.14\\ 12.14 & 299.46 \end{array}\right]. \end{array}$$

In this paper, the threshold method is used to realize simple and fast calculation. It is a commonly used image binarization method. The essence is to use statistical information to determine the segmentation threshold for segmentation. Accurate segmentation of the skin to the image is accomplished by a suitable threshold during this process. We know that different human skin colors can form clusters in the YCrCb space, which provides a basis for skin color segmentation. By creating a skin color model in the YCrCb space, the skin color segmentation is performed using two components, *C*_*b*_ and *C*_*r*_. In this way, the YCrCb space can be obtained by linearly transforming from RGB space, which is simple and fast. Secondly, the *Y* component of the luminance information is removed. At the same time, only two components are included, and the calculation speed is also high. Counting the range of skin to separate the skin from the nonskin area, you get

(10) $$\begin{array}{c} 137<{\text{C}}_{r}<177,\\ 77<{\text{C}}_{b}<127,\\ 190<{\text{C}}_{b}+0.6{\text{C}}_{r}<215. \end{array}$$

### 3.3. Face Recognition Algorithm Based on Linear Subspace

#### 3.3.1. PCA Face Recognition Method

Assuming that there are a total of *M* images in the original image library as training samples, the normalized images are connected by *n* × *n* columns to form a 2*n*-dimensional column vector. Then the original face image vector is represented as X1, X2,…, XM, and the average of the total face image is

(11) $$\begin{array}{c} m=\frac{1}{M}\sum_{i=1}^{M}X_{i}. \end{array}$$

The K-L transform is used to calculate the covariance matrix, also known as the overall dispersion matrix, namely,

(12) $$\begin{array}{c} C=\frac{1}{M}\sum_{i=1}^{M}\left(X_{i}-m\right){\left(X_{i}-m\right)}^{T}=\frac{1}{M}AA^{T}. \end{array}$$

In order to find the eigenvalues of the *n*2 × *n*2 dimensional matrix *C* and the orthogonal normalized eigenvectors *U*, the calculation is too large if the calculation is too large, thus introducing the singular value decomposition theorem (SVD theorem) to solve the problem of high dimensionality. That is, the matrix *R* = AT *A* (*M* × *M* dimensional matrix) is calculated first, and the orthogonal normalized eigenvectors *V* of *R* is calculated, and *U* and *V* have the following relationship:

(13) $$\begin{array}{c} U=AV\Lambda^{-1/2},\\ \Lambda =di\;ag\left(\lambda_{1},\lambda_{2},\ldots ,\lambda_{M-1}\right). \end{array}$$

#### 3.3.2. Fisher Discriminant Analysis Face Recognition Method

*(1) LDA Algorithm*. Assuming that there are a total of *N* images in the original image library as training samples, the normalized image size is *n* × *n*, and the columns are connected to form *n*2 dimensional column vectors. Then the *j*th original face image vector of the *i*-th person is represented as *X*_*ij*_, where *N*_*i*_ indicates that the *N*_*i*_ face image belongs to the *i*-th class, and *C* is the sample class number. The average value of each type of face image is:

(14) $$\begin{array}{c} m_{i}=\frac{1}{N_{i}}\sum_{j=1}^{N_{i}}X_{ij},\;i=1,2,\ldots ,C. \end{array}$$

Defined according to the Fisher guidelines:

(15) $$\begin{array}{c} J\left(W\right)=\underset{w}{\arg\max}\frac{\left|W^{T}S_{b}W\right|}{\left|W^{T}S_{w}W\right|}. \end{array}$$

The optimum projection direction *W* is the value of *W* when the above formula reaches the maximum value. That is, *W* is the solution that satisfies the following equation:

(16) $$\begin{array}{c} S_{b}W_{i}=\lambda_{i}S_{w}W_{i},\;i=1,2,\ldots ,N. \end{array}$$

That is, corresponding to the feature vector corresponding to the larger feature value of the matrix S-1WSb. Note that the matrix has a maximum of only C-1 non-zero eigenvalues, and *C* is the number of categories.

#### 3.3.3. Zero Space Method

Direct linear discriminant analysis (D-LDA) first removes the null space of the interclass dispersion matrix *S*_*b*_, and finds a projection vector to minimize the intraclass dispersion, called D-LDA. The D-LDA method seems to avoid losing the zero space of *S*_*w*_. However, since the ranks of *S*_*b*_ and *S*_*w*_ have such a relationship: *rank*(*S*_*b*_) ≤ *C* − 1 ≤ *rank*(*S*_*w*_) ≤ *N* − *C*, removing the zero space of *S*_*b*_ may result in the loss of part or all of the zero space of *S*_*w*_, which is likely to make *S*_*w*_ full rank, that is, D-LDA indirectly loses *S*_*w*_. Zero space. The zero-space-based LDA first finds the null space of the intraclass dispersion matrix *S*_*w*_, and then projects the original sample onto the zero space of _*w*_*S* to maximize the interclass dispersion matrix *S*_*b*_. The optimal projection vector *W* should satisfy:

(17) $$\begin{array}{c} W^{T}S_{w}W=0,W^{T}S_{b}W\neq 0. \end{array}$$

The optimal discriminant vector *W* should exist in the null space of _*w*_*S*.

### 3.4. Face Recognition Method Based on Kernel Method

#### 3.4.1. KPCA-Based Face Recognition Method

First, the *N* training sample sets X1, X2, X3,…, XN in the original input space RN are nonlinearly mapped to the high-dimensional space by the polynomial kernel function to obtain the kernel matrix of the training set:

(18) $$\begin{array}{c} K_{ij}=K\left(X_{i},X_{j}\right)={\left(\left(X_{i}+X_{j}\right)+1\right)}^{2}. \end{array}$$

Then, the normalized kernel matrix *K* is calculated. Finally, the eigenvalues and eigenvectors of *K* are calculated, and the orthogonal eigenvectors corresponding to the largest *m* eigenvalues are u1, u2, u3,…, um. The sample after projection:

(19) $$\begin{array}{c} y_{j}=\frac{1}{\sqrt{\lambda_{j}}}u_{j}^{T}\left[{\bar{K}}_{1j},{\bar{K}}_{2j},\ldots ,{\bar{K}}_{mj}\right],\;j=1,\ldots ,m. \end{array}$$

The above KPCA feature extraction is completed, and the sample *Y* in the high-dimensional space after the non-linear projection of the face is obtained, and input into the nearest neighbor classifier for classification and recognition.

#### 3.4.2. KFDA-Based Face Recognition Method

First, the N training sample sets X1, X2, X3,…, XN in the original input space RN are nonlinearly mapped to the high-dimensional space by the polynomial kernel function to obtain the kernel matrix of the training set:

(20) $$\begin{array}{c} K_{ij}=K\left(X_{i},X_{j}\right)={\left(\left(X_{i}+X_{j}\right)+1\right)}^{2}. \end{array}$$

After KPCA feature extraction, *Y* is a nonlinear mapping of faces to samples in high-dimensional space. The second feature extraction is performed on *Y* using the LDA algorithm. Calculate the best projection direction *W* according to the Fisher criterion function in the equation, and project *Y* to the optimal projection direction of the LDA.

(21) $$\begin{array}{c} z_{i}=W^{T}y_{i}. \end{array}$$

The above KFDA feature extraction is completed, and *K* is extracted by KPCA and LDA features, and *Z* is input into the nearest neighbor classifier for classification and identification.

#### 3.4.3. KFDA Face Recognition Algorithm Based on Zero Space (KFDA-NULL)

Set in the high-dimensional feature space, the interclass dispersion matrix and the intraclass dispersion matrix of the training samples are *K*_*b*_ and *K*_*w*_, respectively, and the overall dispersion matrix is:

(22) $$\begin{array}{c} K_{t}=K_{w}+K_{b}. \end{array}$$

The total dispersion matrix *K*_*t*_ in the feature space is calculated according to the input spatial data and the kernel function equation; then the eigenvalue analysis is carried out, and the transformation matrix *P*_*k*_ is established by using the eigenvectors corresponding to all nonzero eigenvalues to obtain the intraclass dispersion after the feature space is reduced. Degree matrix and interclass dispersion matrix:

(23) $$\begin{array}{c} {\bar{K}}_{w}=P_{k}^{T}K_{w}P_{k},\\ {\bar{K}}_{b}=P_{k}^{T}K_{b}P_{k}. \end{array}$$

Enter any vector *k*_*j*_=[*k*_1*j*_, *k*_2*j*_,…, *k*_*Nj*_] of the space, and formally project its projection into the high-dimensional feature space.

(24) $$\begin{array}{c} z_{j}=W^{T}k_{j}. \end{array}$$

For large sample problems (*n* < *N*), *S*_*w*_ is full rank and cannot extract any zero space. That is to say, in the case of large samples, any zero space based method fails. However, after nuclear mapping, the zero space based LDA can work on the core sample set. Therefore, for large sample problems, the kernel mapping method is an extension of the zero space method.  Figure 1 is a flowchart of a face recognition system based on multi-feature fusion.

## 4. Experiment

### 4.1. Data Source

The experiments in this paper are mainly based on the public ORL face database and Yale face database. The ORL face database is one of the most widely used face libraries. The database consists of facial expressions and details of black faces on different periods of time. It consists of 40 people, each with 10 front-facing face images of 112 ^∗^ 92 size. Some of them were taken at different times, and the lighting conditions were almost unchanged, most of them were changes in expressions and postures. For example: laughing or not laughing, blinking or closing your eyes, with or without glasses; face posture changes, rotation up to 20 degrees; face size also has up to 10% change. The Yale face library consists of 15 people, each with 11 front-facing faces of 128 ^∗^ 128 size, including different expressions, different lighting, blinking or closing eyes, and wearing and not wearing glasses.

The training set used by Deep ID is Celeb Faces. Deep ID Network Training during the use of this data set, 80% of the data in the training set was used to train the neural network part of the Deep ID network, while the latter Bayesian model was completed by the remaining 20%. Celeb Faces is a large dataset with a total of 87,628 images from 5,436 famous people in the Celeb Faces dataset. This data set is ideally suited for use as a training set and test set for computer vision tasks, and can perform a variety of functions including face detection, facial features, and face recognition.

### 4.2. Experimental Parameter Setting

The AdaBoost training sample library created in this paper has 3000 face samples of 24 × 24 size, including nearly 700 multi-pose face samples with obvious deflection tilt. In the experiment, although the face samples are as much as possible, the face samples will be more good detection results, but at the same time will increase the training burden, so this paper selected 3000 face samples according to the previous detection system. As for the selection of 700 multi-pose faces, it has been better through experiments. Detection, but subsequent algorithm optimization needs to be thoroughly studied and compared. Although the use of skin color segmentation has excluded a large number of nonface background areas, in order to accurately detect the face, a large number of nonface samples are needed for training, so the “bootstrap” method is used to obtain the 5000 background images collected. A large number of non-face samples. The minimum detection rate *m* Din of the strong classifier is set to 0.999, the maximum false detection rate Fmax is 0.5, and the maximum number of training layers is 15.

## 5. Results and Discussions

### 5.1. Analysis of Single Face Recognition Results Based on Skin Color Segmentation

The test results of the single face test set are shown in Table 1:

According to the experimental test results and statistical analysis of the data in Table 1:

The skin color feature is combined with the AdaBoost algorithm to eliminate the complex background of the human face under the gray image, which effectively reduces the false detection rate. However, we also find that the detection rate does not improve after the combination, but has a slight influence. By observing the test results, it was found that the detected image was severely affected by light and other factors, which led to misdetection or damage detected by the AdaBoost method.

As can be seen in Figure 2, the introduction of skin color features into the AdaBoost algorithm is a good limitation of the number of false detection windows, but due to the leak detection of the skin color detection in the test image under weak lighting conditions, it is excluded that the light can be processed by illumination. The face detected by the AdaBoost method, so the skin color + AdaBoost method has more missed faces than the AdaBoost method, but in general, the introduction of skin color features greatly reduces the number of false detection windows, making the skin color + AdaBoost method in ROC The curve performance is better than the AdaBoost method. On this basis, although the method of this paper will also identify some weakly illuminated faces due to the introduction of skin color leakage, but because of the new sparse features instead of Haar features, the AdaBoost method has a better multi-pose face detection effect. Improvement, so that the overall detection efficiency of the algorithm is improved, but also for this reason, the false detection window of this method will be slightly more than the skin color + AdaBoost method.

### 5.2. Analysis of Multi-Face Recognition Results Based on Skin Color Segmentation

The test results of the multi-face test set are shown in Table 2:

By observing Table 2 and the experimental data, we can get the conclusions roughly as shown in Table 1, but compared with Table 1, the false detection rate of the three methods is increased overall, and the detection rate is decreased. This is due to the multi-face image. The background may be more complicated, the face pose is more varied, even occluded and blurred, so the detection effect will be worse than the single face detection. But overall, the skin color + AdaBoost method of this article is still relatively better than the first two methods.  Figure 3 shows the ROC curve for a self-built multi-face test set.

From Figure 3, we can get similar conclusions as shown in Figure 2, but because the background area in the multi-face image is more complicated and the face pose is more diverse, the test performance of the three methods is generally reduced. Overall, the method is still better. In the first two methods, the skin color feature is very good at limiting the false detection rate, and the sparse feature is better for detecting multi-pose faces.

### 5.3. Analysis of Face Recognition Results Based on Linear Subspace

The ORL library consists of 40 people. Each person has 10 different face images. The first 5 images of each person are used as the training set, and the last 5 images are used as test sets. The PCA method is used to select different feature space dimensions and different. The number of samples and the calculation recognition rate are shown in Table 3.

Where *d* is the dimension of the selected sub-space, *n* is the number of selected training samples (3 means 10 out of 10 images for one person, 7 for training), using the most recent neighbor classification. From the experimental data in the table, it is found that as the dimension of the sub-space increases, the recognition rate also increases accordingly. When the dimension of the subspace is small, the increase in the recognition rate is significant. At the same time, the number of training samples also has a great influence on the relationship between the sub-space dimension and the recognition rate. Select the same sub-space dimension, the more training samples, the higher the recognition rate. Therefore, the more samples used for training, the more adequate the training and the better the recognition. Of course, here we have to avoid the situation of training.

When the number of training samples is fixed, the higher the dimension of the sub-space, the higher the recognition rate. Observing a large amount of experimental data, we can see that the maximum value of recognition rate is about *d* = 71 when *n* = 7; the maximum value of recognition rate when *n* = 5 is about *d* = 80; when *n* = 3, the recognition rate The maximum point is around *d* = 90. After that, the sub-space dimension is increased and the recognition rate will not exceed this point. It can be seen that since the PCA method is based on gray scale statistics, some feature vectors may add invalid information such as noise, resulting in a decrease in the recognition rate. When the number of training samples per person is fixed at 5, the ORL face database increases with the dimension of the sub-space, and the changes of the threshold and recognition rate are shown in Figure 4.

When the dimension of the feature sub-space increases, the threshold of the feature value increases, and the recognition rate also increases. When the threshold is 0.65, the corresponding dimension is 12, and the recognition rate tends to be balanced. When the threshold is 0.92, the dimension is 80 and the recognition rate is the highest. In practical applications, the sub-space composed of the feature vectors corresponding to the feature values of 0.8∼0.9 of the overall feature value is generally used for PCA face recognition.

### 5.4. Face Recognition Method Based on Kernel Method

There are 40 people in the ORL, the first 5 images of each person are used for training, the last 5 are used for testing, the nearest neighbor method is used as the classifier, and different kernel functions and corresponding parameters are selected. The recognition results are shown in Table 4.  Table 5 shows the recognition results of different recognition methods in the three databases.

If you choose the polynomial kernel function, you can see from Figure 5 that when *d* = 0.8, KPCA has a higher recognition ability. Therefore, for KPCA, a polynomial kernel function with a small exponent (between 0 and 1) can achieve better recognition. However, for KFDA and zero-space-based KFDA (KFDA + NULL), the recognition rate is the highest when *d* = 2, and KPCA also has a high recognition rate. When the value of *d* is from 0 to 2, the recognition rate of KPCA decreases. KFDA uses LDA for secondary feature extraction based on KPCA feature extraction. When KPCA recognition rate is quite high, it is equal to or close to 100. In the case of %, the secondary feature extraction using LDA will reduce the recognition rate; when the recognition rate of KPCA is relatively low, that is, KPCA cannot extract the discrimination information well, and the secondary feature extraction by LDA can effectively extract the discrimination information, so the recognition rate has increased. When *d* = 2, the recognition rate of KFDA and zero space-based KFDA is the largest. For polynomial functions, in general, *d* = 2.

If the RBF kernel function is selected, *σ*2 = 5 × 106, the above KPCA, KFDA and zero space-based KFDA three face recognition algorithms based on the kernel method have higher recognition ability. From the experimental data in Table 4, it can be concluded that the face recognition algorithm based on the kernel method has good recognition performance when the RBF kernel function is selected and the parameter is set to *σ*2 = 5 × 106.  Figure 6 is a comparison diagram of four face recognition methods based on ICA.

The face is detected by the AdaBoost method, so the skin color + AdaBoost method has more missed faces than the AdaBoost method, but in general, the introduction of the skin color feature greatly reduces the number of false detection windows, making the skin color in the ROC The curve performance of +AdaBoost method is better than that of AdaBoost method. As the dimension of the feature sub-space increases, the threshold of the feature value increases, and the recognition rate also increases. When the threshold is 0.65, the corresponding dimension is 12, and the recognition rate tends to be balanced. When the threshold is 0.92, the dimension is 80, and the recognition rate is the highest. In practical applications, PCA face recognition usually uses a sub-space composed of eigenvectors corresponding to eigenvalues of 0.8 to 0.9 of the total eigenvalues. The three face recognition algorithms based on kernel method, KPCA, KFDA and KFDA based on null space, have high recognition ability. When the RBF kernel function is selected and the parameter is set to *σ*2 = 5 × 106, the face recognition algorithm based on the kernel method has good recognition performance.

## 6. Conclusions

In order to identify and detect human faces through computer vision technology, this paper studies the algorithm and draws the following conclusions:

1. In general, the method used in this paper has improved compared with the traditional AdaBoost method and skin color + AdaBoost method. The introduction of the previous experiment and analysis of skin color features can better eliminate the complex background of non-face. AdaBoost detection is performed compared to directly using grayscale images, which reduces the probability of false detection. In addition, the new sparse features are used to replace the Haar features in the traditional AdaBoost algorithm, so that the system can better cope with the traditional AdaBoost method. Multi-pose face such as deflection tilt effectively reduces the face detection and improves the detection rate, but skin color features and sparse features improve the performance of the system at the same time.
2. Because the self-built face training sample has added the face collected by the laboratory itself, there is a high detection rate in the test. The experiment compares the AdaBoost method, the skin color method and the experimental results of the skin color + AdaBoost method. It can be seen that the method is better than the AdaBoost method in terms of detection rate and false detection rate. At the same time, it is also found that due to the addition of skin color features, it is possible to eliminate the face detected by AdaBoost due to illumination, etc., and the AdaBoost method using a new sparse feature for detecting the face of more gesture modes. It is more likely to cause false detections of complex backgrounds, but also because of the use of skin color features, these false detections are limited to the area of the skin color (such as the hand) background.
3. All operations in the KPCA and KFDA algorithms are performed by the inner product kernel function defined in the original space, and no specific non-linear mapping function is involved. This is the core skill of the nuclear learning method. Zero-space-based KFDA overcomes the effects of illumination and is robust to expression and attitude changes. The zero-space method can overcome the small sample problem in discriminant analysis by finding the best discriminant analysis information existing in the zero space of the interclass dispersion matrix. Combining the zero-space method kernel discriminant analysis method not only improves the ability of discriminant analysis to extract non-linear features, but also overcomes the small sample problem in discriminant analysis.
4. Through the secondary extraction of PCA features, a better recognition result than the PCA method is obtained. These two classical algorithms can be described by the same framework, that is, the corresponding linear feature space is constructed first, then the image is projected to the linear space, and the obtained projection coefficient is used as the identified feature vector. The only difference between the two methods is that the feature space is chosen differently. Aiming at the small sample problem of two linear sub-space methods, PCA and LDA, this paper also proposes a zero-space based Fisher discriminant analysis method. Experiments show that the zero-space-based method makes full use of the zero space in the intraclass dispersion matrix. The useful discriminating information improves the correct rate of face recognition to some extent.

## Figures and Tables

**Figure 1:** Flow chart of face recognition system based on multifeature fusion.

**Figure 2:** Single face test set ROC curve.

**Figure 3:** Self-built multi-face test set ROC curve.

**Figure 4:** PCA recognition rate changes with threshold.

**Figure 5:** Comparison of several face recognition methods on ORL face database (using polynomial kernel function).

**Figure 6:** Comparison of four face recognition methods based on ICA.

**Table 1:** Single face test set test results.

Detection method	Face number	Face detection	Missing face detection	Detection rate	False detection window	False detection rate
AdaBoost	300	275	25	0.917	29	0.097
Color	300	275	28	0.907	14	0.047
Color + AdaBoost	300	287	13	0.957	16	0.053

**Table 2:** Multi-face test set test results.

Detection method	Face number	Face detection	Missing face detection	Detection rate	False detection window	False detection rate
AdaBoost	461	412	49	0.894	57	0.124
Color	461	407	54	0.882	24	0.052
Color + AdaBoost	461	425	36	0.921	29	0.063

**Table 3:** Corresponding recognition rates of different feature sub-space dimensions and number of different training samples in PCA.

Dimension *d*	*N* = 8 (%)	*N* = 7 (%)	*N* = 5 (%)	*N* = 3 (%)
110	96.25	95.83	88	85.71
90	96.25	95.83	88	85.71
80	96.25	96.67	89.5	84.64
71	96.25	96.67	88.5	84.29
31	95	95.83	88.5	81.07
23	95	95.83	87	80.36
17	95	95	83.5	76.07
12	95	95	84	75.71
9	96.25	94.17	84	75.36
6	83.75	84.17	74.5	65

**Table 4:** Identification results when selecting different kernel functions and corresponding parameters on the ORL face database.

ORL face database		KPCA (%)	KFDA (%)	KFDA + NULL (%)
Polynomial kernel function	*d* = 0.8	100	80.5	90.5
	*d* = 0.8	99	84	90.5
	*d* = 0.8	96.5	97	97.5

RBF kernel function	Sig2 = 1.5e8	100	85	92.5
	Sig2 = 5e6	100	98.5	100

**Table 5:** Recognition results of different recognition methods in three databases.

Feature extraction method	Maximum average recognition rate		
	ORL	Yale	Georgia tech
DCT	95.86	83.01	79.99
Gabor	93.78	91.99	69.76
DCT + gabor	95.76	93.02	79.79
DCT + ICA	96.69	92.89	78.36
Gabor + ICA	97.58	96.87	80.29
DCT + gabor + ICA	98.01	95.69	83.98

## Data Availability

No data were used to support this study.

## References

[1] Jiang J., Chen C., Huang K., Cai Z., Hu R. (2016). Noise robust position-patch based face super-resolution via tikhonov regularized neighbor representation. *Information Sciences*.

[2] Crunchant A. S., Egerer M., Loos A. (2020). Automated face detection for occurrence and occupancy estimation in chimpanzees. *American Journal of Primatology*.

[3] Mahmood Z., Haneef O., Muhammad N., Khattak S. (2019). Towards a fully automated car parking system. *IET Intelligent Transport Systems*.

[4] Chrysos G. G., Antonakos E., Snape P., Asthana A., Zafeiriou S. (2016). A comprehensive performance evaluation of deformable face tracking “in-the-wild”. *International Journal of Computer Vision*.

[5] Zhao Q., Ge S. S., Ye M., Liu S., He W. (2016). Learning saliency features for face detection and recognition using multi-task network. *International Journal of Social Robotics*.

[6] Mstafa R. J., Elleithy K. M. (2021). A video steganography algorithm based on kanade-lucas-tomasi tracking algorithm and error correcting codes. *Multimedia Tools and Applications*.

[7] Bong K., Choi S., Kim C., Yoo H. J. (2017). Low-power convolutional neural network processor for a face-recognition system. *IEEE Micro*.

[8] Athanasios V., Nikolaos D., Anastasios D., Eftychios P. (2018). Deep learning for computer vision: a brief review. *Computational Intelligence and Neuroscience*.

[9] Kraus O. Z., Frey B. J. (2016). Computer vision for high content screening. *Critical Reviews in Biochemistry and Molecular Biology*.

[10] Mery D., Svec E., Arias M., Riffo V., Saavedra J. M., Banerjee S. (2017). Modern computer vision techniques for x-ray testing in baggage inspection. *IEEE Transactions on Systems, Man, and Cybernetics: Systems*.

[11] Unger J., Merhof D., Renner S. (2020). Computer vision applied to herbarium specimens of German trees: testing the future utility of the millions of herbarium specimen images for automated identification. *BMC Evolutionary Biology*.

[12] Grys B. T., Lo D. S., Sahin N. (2017). Machine learning and computer vision approaches for phenotypic profiling. *Journal of Cell Biology*.

[13] Gadelmawla E. S. (2021). Computer vision algorithms for measurement and inspection of external screw threads. *Measurement*.

[14] Kovashka A., Russakovsky O., Fei-Fei L., Grauman K. (2016). Crowdsourcing in computer vision. *Foundations and Trends® in Computer Graphics and Vision*.

[15] Du L., Hu H. (2019). Nuclear norm based adapted occlusion dictionary learning for face recognition with occlusion and illumination changes. *Neurocomputing*.

[16] Wu Y., Hu H., Li H. (2019). Age-invariant face recognition using coupled similarity reference coding. *Neural Processing Letters*.

[17] Ergin S., Isik S., Gulmezoglu M. B. (2021). Face recognition by using 2D orthogonal subspace projections. *Traitement du Signal*.

[18] Paithane P. (2021). Framework for AttendanceManagementusing face recognition. *Shanghai Ligong Daxue Xuebao/Journal of University of Shanghai for Science and Technology*.

[19] Nasution M. Z. (2020). Face recognition based feature extraction using principal component analysis (PCA). *Journal of Informatics and Telecommunication Engineering*.

